This article has been retracted.

# Effects of Trace Irrigation at Different Depths on Transcriptome Expression Pattern in Cotton (*G. hirsutum* L.) Leaves

**DOI:** 10.1155/2020/7248513

**Published:** 2020-07-27

**Authors:** Li-yu Chen, Li-feng Zhang, Zhan-yuan Lu, Feng Xian, Jian-zhong Zhang, Yu-chen Cheng, Xiang-qian Zhang, Yan Liu

**Affiliations:** ^1^Hebei Agricultural University, Baoding 071000, China; ^2^Inner Mongolia Academy of Agricultural and Animal Husbandry Sciences, Hohhot 010031, China

## Abstract

Drought is a limiting factor for cotton productivity and quality. Irrigation could increase cotton yield. This study is aimed at formulating a proper irrigation depth for cotton at China' Inner Mongolia and at investigating the molecular mechanism underlying the difference induced by irrigation. Transcriptomic analysis was carried out to reveal the global transcriptome profiles on the leaves of cotton seedlings (*G. hirsutum* L. cv. “Zhongmian 92”) with trace irrigation tapes at 30 cm (D30) and 50 cm (D50) underground. The differentially expressed genes (DEGs) were identified and clustered by functional enrichment analysis. The results showed that no significant differences were found in the lint percentage. The yields of unpinned and lint cotton were increased by the D30 regime but decreased by the D50 regime. Transcriptomic analysis showed that 4,549 nonoverlapped DEGs were identified by comparative analysis. Transcription factors, including *bZIP*, *WARK*, *Myb*, and *NAC*, were altered between D50 and D30. The D50 regime induced more DEGs compared with the D30 regime, which was associated with plant tolerance to abiotic stresses and drought. In conclusion, trace irrigation at 30 cm underground was suitable for cotton irrigation at China's Inner Mongolia, while the D50 irrigation regime influenced the cotton yield via drought stress in cotton plants.

## 1. Introduction

Drought is a major abiotic stress and limiting factor for crop productivity. Global climate changes, especially increased atmospheric temperature and infrequent precipitation, influence the sustainable production of agricultural crops [1, 2]. The amount of irrigation water is positively related to agricultural yield [3]. The yield of wheat, groundnut, soybean, and maize had been reduced to 20.6%, 28.6%, 28.0%, and 39.3%, respectively, from 1980 to 2014/2015 due to drought [3, 4]. The reduction induced by drought stress during the reproductive stage was terrible. The shortage of irrigation water or precipitation has been an enormous threat to world food production.

Plants being stressed with abiotic stresses develop various strategies to survive, including detoxification, adaptability, tolerance, and resistance to stresses. These endogenous strategies continued survival via enhancing tolerance, decreasing sensitivity, and regulating iron balance in plants [5]. For instance, Liu et al. identified 35 transcription factors in cotton under drought stress, including the *Myb*, *WRKY*, and *bZIP* transcription factors (TFs) [6, 7]. TFs serve as participants in plant signal transduction [8]. Transporters, including ATP-binding cassette (*ABC*) transporter, play vital roles in plant development, phytohormone homeostasis, and tolerance and could be induced by abiotic stresses, including heavy metal pollution, salt, and drought stress [9–11]. Huang et al. showed an ABC transporter in rice, *OsALS1*, was positively associated with aluminum tolerance [12]. Also, plant cell membranes perceive stress signals and transduce them by hormone-dependent signaling mechanisms [13]. As reported, MAPK networks are involved in stress response and activate several stress-responsive factors [14]. In stress signaling pathways, calcium (Ca2+) is a universal second messenger, controls many physiological processes in plants. The cytoplasmic Ca2+ concentration varies in response to drought stress and various hormones such as abscisic acid (ABA), jasmonic acid (JA), and ethylene [15]. ABA is a key component in response to various biotic and abiotic stresses. It can modulate large numbers of ABA-responsive genes, which can regulate many physiological processes [16, 17]. Especially in drought stress research, ABA shows extraordinary effects [18–20]. These suggested the magical power of plant tolerance to abiotic stresses.

In addition to plant tolerance, the formulation of suitable irrigation regimes is the most practical solution to hold back the reduction in stress-induced crop production. There is a flood of literature showing the performance and efficiency of different irrigation regimes on improving crop yield and growth [21, 22]. Shao et al. showed that the irrigation treatments of 0% and 40% deficit irrigations with underground pipe depth (60 cm and 80 cm) increased tomato production and fruit quality of total soluble solids, soluble sugar, and vitamin C [22]. Moreover, Falco et al. showed that the seed yield of *Salvia hispanica* L. was increased by irrigation and the antioxidant behavior, contents of *α*-linolenic, and total polyphenolic were decreased with irrigation [21]. These reports suggested that irrigation increased the crop yield and quality reduction by drought.

Cotton (*Gossypium hirsutum* sp.) is a worldwide cultured textile fiber, oil, and livestock feed crop. The worldwide production of cotton is declining due to water deficit [23, 24]. Studies focus on the genomic modified plants having shown the transgenic of tolerance-related genes, including *OsSIZ1* [23], *AtEDT1/HDG11* [25], and *GhAREB/AtABF* [26], increase the increases drought tolerance in cotton. Although genomic modified cotton could increase the yield and tolerance of cotton, proper irrigation regimes showed to be formulated as long-term solutions for rainfed agricultural areas, including China's Inner Mongolia Autonomous Region. Papastylianou et al. showed that irrigation could improve the unginned cotton yield [24]. However, the molecular mechanism in cotton in response to irrigation treatments was still unclear.

It has been reported that the most of the root biomass of crops are in the upper 30 cm of soil [27], and the root density is declined with the water content and soil depth [28, 29]. However, the influence of different irrigation depths on plant growth and yield has not been reported until now as we all know. Cotton roots have strong hydrotaxis and distributed in 0-140 cm of soil depth [30]. Trace irrigation is an irrigation method with strong water-saving ability, which can save more than 70% water than traditional irrigation methods. However, there are still many uncertainties in the application of this irrigation method. In our present study, we investigate the influence of different trace irrigation regimes on cotton yield and molecular features. Cotton plants were irrigated with trace irrigation regimes (dripper depth of 30 cm and 50 cm underground, combined with water amount of 240 m^3^ per 666.67 m^2^). Plant characteristics and yield of unginned and lint cotton were determined. Moreover, we identified the differentially expressed genes (DEGs) altered by different irrigation regimes and analyzed the underlying molecular mechanism of differences induced by different trace irrigation depths. This study would provide us with more basic and specific information on irrigation management for cotton in China's Inner Mongolia Autonomous Region.

## 2. Materials and Methods

### 2.1. Experiment Site

Our experiments were carried out at Dongfeng, Ejina Banner in Alashan League, Inner Mongolia, China (longitude 100°13′E, latitude 40°59′N, about 1000 m above sea level). The climate here is a temperate continental climate with a drought summer. The annual average precipitation from northwest to southeast is from 40 mm to 200 mm; annual average evaporation is from 2400 mm to 4200 mm; the average temperature is 6 ~ 8.5°C. At the initial stage of the test, we measured the content of organic matter (OM), total phosphorus (TP), total nitrogen (TN), total potassium (TK), hydrolysable N (HyN), P2O5, and K2O with three biological repeats for each. The soil physical and chemical properties were measured following the methods described by Bao (Bao, 2000). Briefly, OM content was determined using the potassium dichromate volumetric method; TN was determined by the Kjeldahl method; TP was determined using the sulfuric acid-perchloric acid digestion method; HyN was determined by the alkali-hydrolyzed reduction diffusing method; K2O was determined using the sodium bicarbonate extraction-molybdenum-antimony antispectrophotometric method; P2O5 was determined by the Olsen method. Soil pH was measured with a glass electrode in a 1 : 2.5 soil/water suspension. The crop yields of each plot were recorded quarterly and annually. The details of the physical and chemical characteristics of the soil in the test sites are shown in Table 1.

### 2.2. Plant Material and Experimental Design

Cotton seeds (*G. hirsutum* L. cv. “Zhongmian 92”, strong stress resistance) were purchased from Cotton Institute of Chinese Academy of Agricultural Sciences. All the seeds were sawed in soils' inlaying trace drip irrigation tapes at a depth of 30 cm (D30) and 50 cm (D50) underground in 2016, 2017, and 2018. In total, the experimental field was divided into 9 zones (each experiment was performed in triplicate) according to different drip irrigation depths, and the area of each zone was 30 × 6.15 m (length × width). Irrigation regimes were started in mid-May and ended in late August of each year with continuous trace irrigation. As a supplement, seedlings were drip-irrigated with 66.5 m3 (full irrigation) water per zone for 10-12 days at the beginning of the experiment and for 5-7 days in late July. Rain shelters were used for preventing rainwater during the experimental period. Seedlings drip-irrigated with 66.5 m3 water per zone under the mulching films were used as control material (CK). Each experiment was performed in triplicate. The planting density was 4,800 plants per zone (0.76 m line spacing, 0.1 m individual spacing). Plots were routinely fertilized with base fertilizer (5.5 kg diammonium phosphate and 1.4 kg potassium chlorate per zone) and additional fertilizer (urea 7 kg per zone) and covered with plastic mulch.

### 2.3. Measurements of Growth, Yield and Quality, and Net Photosynthetic Rate (NPR)

Plant characteristics (lint percentage and yields of unginned and lint cotton) were determined in 2016, 2017, and 2018. Also, diurnal changes of NPR in leaves were also measured in 2017 and 2018 according to the method reported previously [31] with a portable LI-6400 photosynthetic gas analysis system (LI-COR, USA) according to the instructions.

### 2.4. RNA Extraction and Sequencing

We used the Illumina-based next-generation sequencing methods to identify the changed gene expression profiles in response to different irrigation treatments. Young leaves were isolated from cotton plants at the flowering and boll setting stage in 2016 with three biological repeats in each group. Total RNA was isolated from leaves using TRIzol (Invitrogen, Carlsbad, CA USA), and DNA fragments were removed using RNase-free DNase I (Takara, Japan). Sample quality was evaluated using Agilent 2100 Bioanalyzer (Agilent Technologies, Carlsbad, CA, USA) and NanoDrop 2000c spectrophotometer (NanoDrop products, Wilmington, DE, USA). The RNA concentration was determined by Qubit Quantification Platform (Life Technologies, Carlsbad, CA, USA). Samples with high quality were subjected to cDNA library construction platform according to standard methods, including RNA fragmentation, double-strand DNA synthesis, adapter appendices, fragment selection, and PCR amplification. The final quality assessment was performed using the Qubit Quantification Platform (Life Technologies) and Agilent 2100 Bioanalyzer (Agilent Technologies). Three cDNA library pools were constructed for each treatment and were loaded on an Illumina HiSeq 4000 sequencing platform.

### 2.5. Data Processing and Transcriptome Analysis

Raw data were obtained using base calling service followed with quality evaluation for the base error rate, Phred score (*Q*_phred_), and GC content. Clean data were obtained by filtering out low-quality reads and adapter sequences in raw data and were then aligned to the *G. raimondii* (https://www.ncbi.nlm.nih.gov/genome/?term=G.%20raimondii) reference genome sequence using the TopHat2 (https://ccb.jhu.edu/software/tophat/index.shtml) [32]. New transcripts were discovered using Cufflinks (v2.1.1, http://cole-trapnell-lab.github.io/cufflinks/) with default parameters [33]; single nucleotide polymorphisms (SNPs) and insertion-deletions (InDels) in clean data were called using GATK2 (v3.2, https://gatk.broadinstitute.org/hc/en-us) with QUAL < 30.0 and QD < 5.0 [34]. The expression levels of transcripts were analyzed using HTSeq software (https://pypi.org/project/HTSeq/) [35], and those with FPKM > 1 were considered expression. Pearson's correlation coefficients (*R*^2^) between samples were calculated for all samples.

### 2.6. Identification and Annotation of DEGs

Transcripts were annotated via BLAST search against the Uniprot/Swiss Prot database. DEGs were called using DESeq analysis [36] and Benjamini-Hochberg (BH) correction (*p* adj < 0.05). DEGs were then subclustered into different clusters using H-cluster, Kmeans, and SOM analysis. Functional annotations of identified DEGs were performed using GOseq analysis [37] (Gene ontology analysis, http://www.geneontology.org/) and Kyoto Encyclopedia of Genes and Genomes (KEGG) Orthology-Based Annotation System (KOBAS) server (http://kobas.cbi.pku.edu.cn/home.do) [38] with corrected *p* value (*p* adj) < 0.05. TFs among identified DEGs were recognized using iTAK (v1.2) with default parameters [39].

### 2.7. Statistical Analyses

Statistical analyses of all data (mean ± standard deviation) were analyzed using SPSS 17.0. Differences between two groups were analyzed using Student *t*-tests, and significances among groups were identified using one-way ANOVA. *p* value < 0.05 was considered statistically significant.

## 3. Results

### 3.1. Different Irrigation Regimes Affect Cotton Yield and NPR

The irrigation depth did not significantly influence the lint percentage according to these three years of data in Table 2.

In 2017, the unginned cotton yield decreased with the irrigation depth: CK > D30 > D50. As for the yield of lint cotton, there were similar trends to unginned cotton yield. Similarly, D30 had the highest lint cotton yield, and CK had the least in 2016 and 2018. Also, the lint cotton yield in 2017 showed the same trend among different groups as unginned cotton yield. These data suggested that the “Zhongmian 92” cotton yield was significantly affected by different irrigation depths. The dynamic change of NPR in 2017 and 2018 presented double peak curves, and the peak value appeared at 10 : 00 and 14 : 00, respectively (Figures 1(a) and 1(b)).

The NPR of all treatments decreased at 12 : 00. The diurnal variation of NPR in two years showed that the effects of different treatments could be divided into three trends: the straight-up period (6 : 00-10 : 00), moderate fluctuation period (decline at 10 : 00~12 : 00 and rise at 12 : 00-14 : 00), and significant decline period (18 : 00-20 : 00). The order of dynamic change of NPR in different groups was D30>D50>CK. The effect of different trace irrigation depths on NPR was visible. The higher NPR in D30 was in line with the increased cotton yield. The NPR results also provided evidence that 30 cm was appropriate for trace irrigation.

### 3.2. Summary and Elevation of Illumina HiSeq Sequencing Data

In order to investigate the underlying molecular mechanisms responsible for the difference in cotton yield induced by different irrigation regimes, we conducted the Illumina transcriptome sequencing on *G. hirsutum* L. cv. “Zhongmian 92” cotton leaves. Illumina HiSeq 4000 sequencing produced average clean bases of 7.3 Gb for each sample, with an average *Q*_30_ value of 94.11%, GC content of 43.39%, and 88.92% mapping ratio to *G. raimondii* reference genome sequence (Supplementary Table S1). Clean reads totally contained 64,362 transcripts (6,414 novel and 57,948 known transcripts), 641,982 SNPs (average of 71,331), and 186,145 InDels (average of 20,683; Table S1). Among known transcripts, 41.92%~44.91%, transcripts had FPKM values of <1 (no expression). The FPKM density distribution is shown in Supplementary Figure S1A. Pearson's correlation coefficients (*R*^2^) between samples were higher than 0.9 (0.924~ 1; Supplementary Figure S1B).

These results suggested the high quality and consistency of the next-generation sequencing data from cotton leaves.

### 3.3. Identification and Annotation of DEGs in Cotton in Response to Different Irrigation Regimes

A total of 2008 and 4050 DEGs (4555 non-overlapped DEGs) were identified in cotton in response to irrigation regime at 30 cm and 50 cm compared with control treatment (DESeq analysis with BH correction *p* adj < 0.05; Figures 2(a) and 2(b)).

A total of 4549 nonoverlapped DEGs were identified through pairwise comparison and were classified into 6 H-clusters according to the expression profiles (Figure 2(c)). In total, D50 induced a number of DEGs related to plant defense, tolerance, and stress response as well as in growth and development.

### 3.4. Identification of DEG Regulated to Plant Defense, Tolerance, and Stress Response

Among these DEGs, a large number of genes encoding the members of tolerance associated factors were identified.  Figure 3 shows the number of upregulated DEGs encoding serine and/or threonine-protein kinases (including CBL-interacting serine/threonine-protein kinase (*CIPK*)1, *CIPK3/5/9/11*, serine/threonine-protein kinase RLCKVII, and receptor-like serine/threonine-protein kinase ALE2), ABC transporters (like upregulated *ABCC3*, *ABCG36*, and *ABCG29* genes and downregulated *ABCI19*, *ABCB1*, *ABCC8*, and *ABCB8* genes), *NAC* transcription factors, nucleobase-ascorbate transporters (*NATs*; like *NAT3*, *NAT6*, and *NAT11*), zinc finger proteins, cytochrome P450 enzymes, dehydration-responsive proteins, and bZIP proteins is higher in cotton plants in response to D50 irrigation depth than D30. In addition, the number of downregulated DEGs encoding *Myb* transcription factors, oxide-related proteins, cinnamyl-alcohol dehydrogenase (*CAD*), NADP-dependent enzymes, photosystem II proteins, and UDP-glycosyltransferases (*UDPGs*) in the plant with D50 treatment is higher than D30 treatment (Figure 3).

### 3.5. Identification of DEGs Related to Plant Growth

We also found that some genes related to metabolism and growth in plants were downregulated by D30 and D50 irrigation regimes, including *CAD* (*CAD1*, probable *CAD9*, and zinc-binding alcohol dehydrogenase domain-containing protein 2 (*ZADH2*)), UDP-glycosyltransferases (including UDP-glycosyltransferase 90A1 (*UGT90A1*), *UGT74E2*, and *UGT92A1*), NADP-dependent enzymes (including NADP-dependent glyceraldehyde-3-phosphate dehydrogenase GAPN and NADP-dependent malic enzyme 4, chloroplastic (*NADP-ME4*)), and photosystem II proteins (photosystem II repair protein PSB27-H1, photosystem II reaction center W protein, and chloroplastic (PsbW), and photosystem II reaction center PSB28 protein, chloroplastic (*PSB28*)). We found most of these DEGs were downregulated in D50 versus CK and/or D30 versus CK (Figure 3).

### 3.6. Identification of TFs among DEGs

Overall, 335 TFs belonging to 56 families (Supplementary Table S2 and Figure 3) were identified from the DEGs. The abundant TF families, including 34 *Myb*, 14 *WRKY*, 14 *NAC*, 7 Tubby-like F-box proteins (*TUBs*), 13 basic helix-loop-helix (*bHLH*), 10 *bZIP*, 9 Auxin/*IAA*, 9 *MADS*, and 11 *GRAS* were dysregulated by both D30 and D50 irrigation regimes. More numbers of dysregulated TFs were observed in plants with the D50 irrigation regime than the D30 regime. In our present study, a total of 44 zinc finger proteins, including C2C2-Dof, C2H2, orphans type, C3H, and C2C2-CO-like, were identified in DEGs induced by D30 and D50 regimes.

### 3.7. Annotation of DEGs Induced by D30 and D50 Irrigation Regimes

Based on the DEGs, respectively, induced by D30 and D50 irrigation regimes, GO enrichment analysis showed DEGs by D30 versus CK were associated with 13 biological processes (Supplementary Table S3), while that by D50 versus CK was involved in 100 biological processes (Supplementary Table S4) significantly (*p* adj < 0.05). That was true for the KEGG pathway enrichment analysis for DEGs by D30 versus CK (8 pathways; Supplementary Table S5) and D50 versus CK (20 pathways; Supplementary Table S6). DEGs induced by the D30 irrigation regime was associated with flavonoid biosynthesis, biosynthesis of secondary metabolites, Vitamin B6 metabolism, and glyoxylate and dicarboxylate metabolism (Supplementary Table S5), while those induced by the D50 irrigation regime were also enriched into other pathways like thiamine metabolism, butanoate metabolism, ascorbate, and alternate metabolism, pentose phosphate pathway and sulfur metabolism besides the pathways mentioned above (Supplementary Table S6). These differences revealed that D30 and D50 irrigation regimes had different influences on cotton plants, which might be responsible for the difference in cotton yield.

### 3.8. DEGs between D30 and D50 Irrigation Regimes

We compared the DEGs between D30 and D50 irrigation regimes and revealed that only 109 DEGs are there between them, including 83 downregulated DEGs and 26 upregulated DEGs (Figure 4(a) and Supplementary Table S7).

Among the downregulated DEGs, including ABCG22, cytokinin dehydrogenase 5 (*CKX5*), *CKX7*, heat stress transcription factor (*HSTF*) A-6b, Shikimate O-hydroxycinnamoyltransferase (*HCT*), *CYP71A1*, and *WRKY70* were identified, while some genes, including caffeoylshikimate esterase gene (*CSE*) and leucoanthocyanidin reductase gene (LR), were downregulated in the D50 group. Only one significant KEGG pathway “Flavonoid biosynthesis” (involving *CYP71A1* and *HCT*) was annotated (*p* adj < 0.05). Among the top 10 pathways, the zeatin biosynthesis (downregulated *CKX5* and *CKX7*), galactose metabolism (downregulated phosphoglucomutase (*PGM*)), and pentose phosphate pathways (downregulated NADP-dependent glyceraldehyde-3-phosphate dehydrogenase and *PGM*) were identified. The top 20 KEGG pathways associated with the DEGs by D50 versus D30 are shown in Figure 4(b).

## 4. Discussion

Our present study demonstrated that the irrigation depth influences the yield of cotton. The irrigation at 50 cm depth significantly reduced the yield in comparison with the 30 cm irrigation depth. For the 30 cm irrigation depth, the yields of unginned and lint cotton were higher than those in the 50 cm depth, which indicated that 30 cm might be an appropriate trace irrigation depth. In addition, the fact that the 50 cm irrigation regime induced more DEGs associated with the plant tolerance and defense might show that the 50 cm irrigation caused stress to the cotton plant.

### 4.1. Influence of Irrigation Depth on Plant

Fan et al. have reported that more than half of the root biomass of wheat, maize, oat, barley, pea, chickpea, soybean, and canola is in the upper 30 cm of soil [27]. Aggarwal et al. [28] and Zhao et al. [29] showed that the vertical depth of 45 cm contained >95% of cotton roots. The root density is declined with the water content in soil [28, 29]. The irrigation at 30 cm depth covered the root system of cotton, while that at the 50 cm depth might results in a drought status for the upper root system due to the leakage. This hypothesis was in line with the increased number of DEGs associated with plant tolerance and defense induced by the D50 irrigation regime. In combination, the fact that the higher NPR by D30 compared with the D50 irrigation regime showed that the D30 irrigation regime was suitable for improving the cotton yield.

### 4.2. TFs among DEGs Related to Plant Defense and Tolerance

TFs play vital and essential roles in plant development, resistance, and tolerance to various stresses. We identified a total of 335 TFs belonging to 56 families among the DEGs induced by D30 and D50 irrigation regimes. For instance, *WRKY33* from wheat is a drought-responsive factor conferring drought resistance in *Arabidopsis* [40]; *WRKY41* and *WRKY17* from cotton positively regulated drought tolerance in *Nicotiana benthamiana* [41, 42]. Mao et al. revealed that there were 30 *bHLH* factors which responded to drought and/or salt stress in apple (*Malus domestica* Borkh.) [43]. Liu et al. identified that there were 7 *Myb*, 16 *WRKY*, 14 *bHLH*, and 14 *bZIP* TFs in cotton under drought stress conditions [6]. Zinc finger proteins regulate plant tolerance to abiotic and biotic stresses, including salt, iron toxicity, and drought [44–47]. A total of 44 zinc finger proteins including C2C2-Dof, C2H2, orphan type, C3H, and C2C2-CO-like were induced by D30 and D50 regimes.

With enrichment analysis, we observed that these TFs were enriched into terms of metabolic processes and component of membrane, regulatory activity, and protein binding, which were involved in pathways including “circadian rhythm” (ath04712), and “plant hormone signal transduction” (ath04075), revealing the essential roles of these transcription factors in plant development and responses. Compared with the D30 regime, more TFs were observed in plants with the D50 regime, and they were enriched into more KEGG pathways by controlling the metabolic processes of organic acid, steroid, and pyruvate. These results suggested that the D50 regime is not suitable for cotton irrigation management.

### 4.3. ABC Transporters in Response to Irrigation Regimes

Among the DEGs, we identified several transporter families that were enriched, including *ABC* and *NAT* transporters. *ABC* transporters are primary pumps in membranes mediating the uptake of iron, phytohormones, molecular substrates, and nutrients [48–51]. These transporters confer plant tolerance. *AtABCG29* serves as a monolignol transporter in the biosynthesis of lignin [9]; *AtABCG36* confers auxin homeostasis in *Arabidopsis* [11]; *AtABCB1*, *AtABCB9*, and *AtABCB11* act as auxin exporters in *Arabidopsis* [52–54]. Some ABC transporters were involved in drought tolerance, including *AtABCG25* [10] and *AtMRP4* [55], by regulating water transpiration and stomatal opening. *Arabidopsis* ABC transporter C family member 16 (*AtABCG16*) was induced by ABA and bacterial infection [56]. Moreover, *Arabidopsis thaliana* and rice seedlings overexpressing *AtABCC3* and *OsALS1* had enhanced tolerance to cadmium [57] and aluminum toxicity [5], respectively; knockout of *OsALS1* in rice resulted in increased sensitivity to aluminum [12]. In our study, we identified several ABC transporter encoding genes, including upregulated *ABCC3*, *ABCG36*, and *ABCG29* genes and downregulated *ABCI19*, *ABCB1*, *ABCC8*, and *ABCB8* genes, by trace irrigation at 30 cm and 50 cm depths. These suggested the potential roles of these ABC transporters for detoxification of iron toxicity and regulating water use in plants.

### 4.4. NAT Transporters in Response to Irrigations

The *NAT* family consists of a larger number of functional redundant members [58]. The functions of *NAT* family members in plant tolerance are rarely reported. Sun et al. identified that there are 14 *NAT* members in apple (*Malus domestica*), and MdNAT6/3/11 were significantly induced by drought conditions [58]. In our present study, we found that trace irrigation at the 50 cm depth increased the expression of three *NAT* genes (*NAT3*, *NAT6*, and *NAT11*), and irrigation at the 30 cm depth only upregulated *NAT6* comparing with control conditions. These NAT members were annotated into the same GO terms with ABC transporters. These differences suggested that NATs were proved responsive to both droughts and might have potential roles in detoxification of iron toxicity and regulating water use in cotton plants. The higher number of downregulated ABC transporters and upregulated NAT transporters by the D50 regime showed that it caused drought-like stresses in cotton. Previous studies reported that the NAT family highlighted the importance of the first amino acid position of the motif in the definition of substrate specificity [59–61]. Verónica et al. identified 12 AtNATs in Arabidopsis thaliana, which play roles in abiotic stress [62]. These evidences suggest that NAT may play a similar role in cotton.

### 4.5. DEGs Related to Plant Growth

We also found that some genes related to metabolism and growth in plants were downregulated by the D50 irrigation regime, including *CAD1*, *UGT90A1*, *UGT74E2*, *UGT92A1*, *GAPN*, *PsbW*, and *PSB28. UGT74E2* was involved in water stress response in *Arabidopsis* plant through its activity to auxin indole-3-butyric acid (*IBA*) [63]; GapN catalyzes the oxidation of glyceraldehyde 3-phosphate to 3-phosphoglycerate and is an alternative *NADPH* source [64, 65]; *PsbW* and *PSB28* are involved in the stabilization and recovery of photosystem II complexes, respectively [66, 67]. The downregulation of these genes in response to the D50 irrigation regime compared with the D30 irrigation regime might reveal the disturbance of photosystem II systems and the energy source by the D50 regime.

In addition, we identified the downregulated DEGs by D50 versus D30 including *CKX5* and *CKX9*, which was related to Zeatin biosynthesis and *HCT* to “flavonoid biosynthesis”. *CKXs* control the degradation of the plant hormone cytokinin [68]. The downregulated *CKX5* and *CKX9* by the D50 regime versus the D30 regime might show the inhibition of the degradation of plant cytokinins, which control the growth and devolvement of plants. Previous reports showed that elevated cytokinin might promote drought tolerance [69]. *HCT* links flavonoid biosynthesis and the lignin/monolignol pathway [70]. The expression of *HCT* could be downregulated by the exogenous *CPPU* and therefore blocking the synthesis of anthocyanin but was increased by ABA and thus enhancing the accumulation of anthocyanin in *Litchi chinensis* pericarp [71]. The downregulation of these genes by the D50 regime compared with the D30 regime showed that a D50 irrigation regime caused growth inhibition and stresses.

## 5. Conclusion

In summary, we found that different trace irrigation regimes influence cotton yield and plant responses. However, trace irrigation at the 50 cm depth induced a lower yield of unginned and lint cotton in comparison with irrigation at the 30 cm depth. The results show that a deeper irrigation depth will induce more transcription factors in response to drought stress, indicating that 50 cm is not a good depth of trace irrigation in cotton. NAT family members, ABC transporters, and transcription factors (TFs) play important roles in cotton in response to drought stress, indicating that the response of cotton to drought stress is a complex process. An irrigation depth of 30 cm showed a good effect, which might be closely related to the length of cotton root system and growth ability. In short, trace irrigation can greatly save irrigation water greatly, but different irrigation depths have different impacts on plants.

## Figures and Tables

**Figure 1:** The NPR measurement. (a) and (b) Show the NPR results in 2017 and 2018, respectively. The *x*-axis represents time, and the *y*-axis represents NPR values. Different types of lines represent different groups.

**Figure 2:** The profiles of differentially expressed genes (DEGs) in response to different irrigation regimes. (a) Volcanic map and of differentially expressed genes (DEGs). (b) Venn analysis results between D30 vs. CK and D50 vs. CK. (c) Heatmap representation of the expression profiles of the DEGs. The redder the square color, the higher the gene expression level.

**Figure 3:** The number of genes encoding related factors in cotton plants.

**Figure 4:** The differentially expressed genes (DEGs) between D50 and D30 irrigation regimes. (a) Shows the volcanic map of DEGs between D50 and D30. (b) Shows the results of KEGG pathway enrichment analysis.

**Table 1:** The physical and chemical characteristics of the soil in the test sites.

Characteristics	Organic matter (g/kg)	Total *N* (g/kg)	Total *P* (g/kg)	Total *K* (g/kg)	Hydrolysable *N* (mg/kg)	P_2_O_5_ (mg/kg)	K_2_O (mg/kg)	pH
Value	12.21	0.58	0.32	20.27	49	10.87	149.17	8.49

**Table 2:** The indicators of cotton plant growth, yield, and quality in different irrigation regimes.

Year	Groups	Lint P. (%)	Unginned Y. (kg/hm^2^)	Lint Y. (kg/hm^2^)
2016	CK	41.30 ± 0.32	5501.14 ± 57.21b	2410.5 ± 22.20c
	D30	43.80 ± 0.51	5886.47 ± 69.92a	2799.88 ± 39.33a
	D50	44.28 ± 1.13	5550.05 ± 56.67b	2505.33 ± 24.18b
2017	CK	41.94 ± 1.23	5557.67 ± 56.91a	2290.20 ± 24.23a
	D30	43.72 ± 0.63	5244.15 ± 56.91b	2202.75 ± 25.02b
	D50	45.04 ± 0.76	4445.85 ± 63.95c	1852.50 ± 26.46c
2018	CK	41.94 ± 1.23	5557.20 ± 56.91c	2290.20 ± 24.23c
	D30	43.38 ± 1.08	6224.40 ± 51.99a	2706.30 ± 23.33a
	D50	44.51 ± 0.96	5850.75 ± 68.07b	2585.10 ± 29.56b

## Data Availability

We submitted the data in supplementary files to ensure that others can see and share it.

## Supplementary Materials

Supplementary Materials Figure S1 Pearson correlation between samples. Table S1: the summary of Illumina HiSeq sequencing for *Gossypium hirsutum* L. cv. Zhongmian 92. Table S2: the transcription factor among the differentially expressed genes identified in our study. Table S3: the GO terms of differentially expressed genes in the D30 irrigation regime comparing with control treatment. Table S4: the GO terms of differentially expressed genes in the D50 irrigation regime comparing with control treatment. Table S5: the KEGG pathways of differentially expressed genes in the D30 irrigation regime comparing with control treatment. Table S6: the KEGG pathways of differentially expressed genes in the D50 irrigation regime comparing with control treatment. Table S7: the list of the differentially expressed genes by D50 versus D30.
